# Association between General Anesthesia and the Occurrence of Cerebrovascular Accidents in Hip Fracture Patients

**DOI:** 10.1155/2021/7271136

**Published:** 2021-12-18

**Authors:** Hu Wang, Lingyan Gao

**Affiliations:** ^1^Department of Emergency Surgery, The Fifth People's Hospital of Jinan, Jinan 250022, Shandong Province, China; ^2^Department of Anesthesiology, Pingyi County People's Hospital, Linyi 273300, Shandong Province, China

## Abstract

**Background:**

General anesthesia is an important factor leading to postoperative complications, and cerebrovascular accidents take the first place in the causes of postoperative death. Therefore, it is extremely important to explore the correlation between general anesthesia and the occurrence of cerebrovascular accidents in hip fracture patients.

**Objective:**

To explore the association between general anesthesia and the occurrence of cerebrovascular accidents in hip fracture patients.

**Methods:**

The data of 240 hip fracture patients treated in our hospital from February 2017 to February 2021 were retrospectively analyzed, and the patients were divided into the general anesthesia group (*n* = 120) and nongeneral anesthesia group (*n* = 120) according to whether or not they received general anesthesia, so as to compare their incidence rate of cerebrovascular accidents between the two groups, record their hemodynamic changes, and analyze the association between various risk factors under general anesthesia and the occurrence of cerebrovascular accidents.

**Results:**

No statistical differences in patients' general information such as age and gender between the two groups were observed (*P* > 0.05); compared with the nongeneral anesthesia group, the incidence rate of cerebrovascular accidents was significantly higher in the general anesthesia group (*P* < 0.001); between the two groups, the heart rates and mean arterial pressure (MAP) at 15 min after anesthesia, at the time of skin incision, and 15 min before the end of surgery were significantly different (*P* < 0.05); according to the multiple logistic regression analysis, general anesthesia was a risk factor affecting the occurrence of cerebrovascular accidents in hip fracture patients, and under general anesthesia, age ≥80 years, BMI ≥23 kg/m^2^, types of anesthetic drugs ≥4, intraoperative blood pressure ≥140 mmHg, and intraoperative heart rate ≥80 bpm were also regarded as the risk factors.

**Conclusion:**

General anesthesia is a risk factor affecting the occurrence of cerebrovascular accidents in hip fracture patients, and under general anesthesia, age ≥80 years, BMI ≥23 kg/m^2^, types of anesthetic drugs ≥4, intraoperative blood pressure ≥140 mmHg, and intraoperative heart rate ≥80 bpm will further increase the possibility of cerebrovascular accidents.

## 1. Introduction

The hip joint is an important joint connecting the trunk and lower extremities and is composed of the acetabulum, femoral head, articular capsule, and ligaments, which mainly serves to carry the weight of the body and accomplish the motor function in multiple axial directions. With increasing age, the hip joint undergoes gradual wear, which, combined with the decreasing fracture resistance capacity of the elderly, leads to high incidence of hip fracture [1–3]. According to a World Health Organization survey report, 30.0% of hip fractures worldwide occur in China [4], and surgery is the preferred treatment modality for patients without surgical contraindications, but 32.3% of patients will experience perioperative complications, with a probability of dying from complications reaching 30.0% 1 year after surgery and risk of death lasting for up to 10 years [5–7]. Among all the causes of postoperative death in patients with hip fracture, cerebrovascular accidents take the first place, so it is extremely important to explore the risk factors that induce cerebrovascular accidents. In practice, most hip fracture patients are aged and usually have underlying diseases and poor tolerance for anesthesia and surgery, and the cerebral vasoconstrictor anesthetic drugs will further increase their cerebrovascular resistance and lead to cerebral blood flow and metabolic rate decline [8], easily resulting in severe central nervous system (CNS) complications, so there is a close relationship between general anesthesia and cerebrovascular accidents. Some studies have confirmed that general anesthesia is a risk factor for the occurrence of cerebrovascular accidents [9, 10], but no research has deeply explored the correlation of the occurrence of cerebrovascular accidents with general anesthesia, and the effects of factors such as blood pressure, age, and the amount of medications on the incidence of cerebrovascular accidents in hip fracture patients under general anesthesia remain unclear. Based on this, 240 hip fracture patients were selected for the study herein, with the results reported as follows.

## 2. Data and Methods

### 2.1. Study Design

This study was a retrospective study and conducted in our hospital from February 2017 to February 2021 to explore the association between general anesthesia and the occurrence of cerebrovascular accidents in hip fracture patients. It was a double-blind study, meaning that neither the study subjects nor the researchers were aware of trial grouping, and the study designer was responsible for arranging and controlling the full trial.

### 2.2. Recruitment of Research Objects

The data of hip fracture patients treated in our hospital from February 2017 to February 2021 were retrospectively analyzed, and the patients were recruited according to the following inclusion and exclusion criteria.

#### 2.2.1. Inclusion Criteria

The inclusion criteria were as follows: (1) the patients were diagnosed with hip fracture for the first time after CT examination [11], and their results of routine blood test and urinalysis, electrocardiogram (ECG), and ultrasonic examination met the surgical indications; (2) the patients were treated in our hospital the whole time and did not transfer to another hospital or stop the treatment; (3) the patients had complete clinical data; and (4) the patients' American Society of Anaesthesiologists (ASA) grade was I-II [12].

#### 2.2.2. Exclusion Criteria

The exclusion criteria were as follows: (1) the patients could not communicate with others due to hearing disorders, language disorders, unconsciousness, mental diseases, or other factors; (2) the patients quit the treatment or changed the treatment regimen during the study; (3) the patients had other severe organic diseases; (4) the patients had fracture of other parts or pathological fracture; (5) the patients had systemic infectious diseases; (6) the patients had contraindications of surgery or general anesthesia; and (7) the patients took sedative and analgesic drugs for a long time.

### 2.3. Steps

A total of 240 hip fracture patients were included in the study and divided into the general anesthesia group (*n* = 120) and nongeneral anesthesia group (*n* = 120) according to whether or not they accepted general anesthesia. On the day that the patients agreed to join the study, the study team collected the sociodemographic data and clinical performance data and, after surgery, recorded the number of patients with cerebrovascular accidents and analyzed the correlation of general anesthesia with the occurrence of cerebrovascular accidents.

### 2.4. Moral Consideration

The study met the principles in the World Medical Association Declaration of Helsinki [13] and was approved by the review committee of the hospital ethics review organization. After recruitment, the study team explained the study purpose, meaning, content, and confidentiality to the patients and asked the patients to sign informed consent.

### 2.5. Criteria of Quitting the Trial

For patients who had one of the following situations and were judged as unsuitable for continuously accepting the trial by the study team, their case record forms would be reserved but not used for data analysis: (1) occurrence of adverse events or serious adverse events; (2) condition worsening during the trial; (3) occurrence of certain serious comorbidities or complications; (4) unwilling to proceed the clinical trial and proposing the demand of quitting the clinical trial to the study team.

### 2.6. Methods

By means of retrospective analysis, the patients' medical records from February 2017 to February 2021 were consulted, and their data including gender, age, BMI, mean body mass, marital status, place of residence, monthly income, educational degree, living habits, complications, and history of cerebrovascular accidents were collected; through the observation of the incidence of cerebrovascular accidents during the perioperative period, the association between risk factors such as general anesthesia and the occurrence of cerebrovascular accidents was analyzed by multiple logistic regression (step-by-step method).

### 2.7. Observation Criteria

1. General information: the general information extract form was established by the patients themselves, covering gender, age, BMI, mean body mass, marital status, place of residence, monthly income, educational degree, living habits, complications, and history of cerebrovascular accidents
2. Incidence of cerebrovascular accidents: the diagnosis basis of cerebrovascular accidents was relevant standards in *Internal Medicine* (8^th^ edition) [14], and the patients should be diagnosed by brain CT and MRI
3. Changes in hemodynamics: all patients received the tests of perioperative mean arterial pressure (MAP) and heart rate (HR), after entering the operating room, left radial artery cannulation was performed for pressure measurement, and before anesthesia (*T*_1_), 15 min after anesthesia (*T*_2_), at the time of skin incision (*T*_3_), and 15 min before the end of surgery (*T*_4_), the patients' MAP, HR, and saturated pulse oxygen (SpO_2_) were recorded and compared
4. Association between various risk factors under general anesthesia and the occurrence of cerebrovascular accidents: the association between general anesthesia and the occurrence of cerebrovascular accidents as well as between factors under general anesthesia including age, BMI, number of anesthetic drugs, intraoperative blood pressure, and HP and the occurrence of cerebrovascular accidents was analyzed

### 2.8. Statistical Processing

In this study, data processing software was SPSS 20.0, picture drawing software was GraphPad Prism 7 (GraphPad Software, San Diego, USA), the patients' general information included enumeration data and measurement data, the incidence of cerebrovascular accidents included enumeration data, and the hemodynamic indicators included measurement data. The data in this study included enumeration data (tested by *X*^2^ test) and measurement data (tested by *t*-test), and differences were considered statistically significant at *P* < 0.05. Taking the occurrence of cerebrovascular accidents as the dependent variable and general anesthesia as the independent variable, the correlation of general anesthesia with the incidence of cerebrovascular accidents as well as that of age, BMI, number of anesthetic drugs, intraoperative blood pressure, and HR under general anesthesia with the incidence of cerebrovascular accidents was analyzed by multiple logistic regression (step-by-step method).

## 3. Results

### 3.1. Comparison of Patients' General Information

No statistical differences in patients' general information between the two groups were observed (*P* > 0.05). See Table 1.

### 3.2. Comparison of Incidence Rates of Cerebrovascular Accidents in Patients

The incidence rate of cerebrovascular accidents was significantly higher in the general anesthesia group than the nongeneral anesthesia group (*P* < 0.001). See Figure 1.

### 3.3. Comparison of Changes in Patients' Hemodynamic Indicators

At *T*_1_, *T*_2_, *T*_3_, and *T*_4_, the HP and MAP were significantly different between the two groups (*P* < 0.05). See Figure 2.

Figure 2(a) shows the HR. At *T*_1_, no statistical difference in HR between the two groups was observed (73.65 ± 5.68 vs. 73.68 ± 5.54, *P* > 0.05); and at *T*_2_, *T*_3_, and *T*_4_, the HR of the general anesthesia group was significantly different from that of the nongeneral anesthesia group (82.65 ± 5.10 vs. 70.65 ± 5.58, 85.98 ± 5.65 vs. 71.66 ± 5.20, and 70.65 ± 5.10 vs. 72.12 ± 5.99, *P* < 0.05).

Figure 2(b) shows the MAP. At *T*_1_, no statistical difference in MAP between the two groups was observed (13.11 ± 0.54 vs. 13.13 ± 0.58, *P* > 0.05); and at *T*_2_, *T*_3_, and *T*_4_, the MAP of the general anesthesia group was significantly lower than that of the nongeneral anesthesia group (12.30 ± 0.54 vs. 12.98 ± 0.42, 12.05 ± 0.32 vs. 12.87 ± 0.65, and 11.87 ± 0.35 vs. 12.68 ± 0.40, *P* < 0.001).

Figure 2(c) shows SpO_2_. At *T*_1_, *T*_2_, *T*_3_, and *T*_4_, no statistical differences in SpO_2_ between the two groups were observed (93.98 ± 1.23 vs. 93.97 ± 1.26, 99.65 ± 1.30 vs. 99.64 ± 1.20, 99.42 ± 1.65 vs. 99.46 ± 1.35, and 98.96 ± 1.35 vs. 99.05 ± 1.23, *P* > 0.05).

### 3.4. Association between Various Risk Factors under General Anesthesia and the Occurrence of Cerebrovascular Accidents

According to the multiple logistic regression, general anesthesia was a risk factor affecting the occurrence of cerebrovascular accidents in hip fracture patients, and under general anesthesia, age ≥80 years, BMI ≥23 kg/m^2^, number of anesthetic drugs ≥4, intraoperative blood pressure ≥140 mmHg, and intraoperative heart rate ≥80 bpm were also related. See Tables 2 and 3.

## 4. Discussion

Hip fracture is an important complication of osteoporosis, which mainly includes femoral neck fracture and intertrochanteric fracture, and is commonly found in the elderly. After fracture, the mortality rate can reach 50.0%, and the 5-year survival rate is only 20.0% [15, 16], indicating poor prognosis of the disease. In current practice, surgery is advocated for patients without surgical contraindications because according to the clinical data, nonsurgical treatment will further elevate patient mortality [17, 18], while surgery can shorten patients' bed time and accelerate their limb recovery. However, elderly patients with hip fracture usually have poor body tolerance and a high rate of perioperative complications, among which cerebrovascular accidents are one of the most serious ones and also the leading cause of postoperative death [19]. Studies have shown many risk factors affecting cerebrovascular accidents, and currently, the well-established ones include history of cerebrovascular accidents, history of hypertension, general anesthesia, anesthetic drug dosage, and intraoperative blood pressure [20, 21], in which general anesthesia is closely related to factors such as anesthetic drug dosage and intraoperative blood pressure, and therefore, it may be one of the most critical elements affecting cerebrovascular accidents.

General anesthesia is the main type of anesthesia for hip fracture patients, and usually, 3-4 kinds of drugs are applied, which will reduce the tension of the patients' peripheral blood vessels and their cardiac output and then cause fall of blood pressure and insufficient cerebral perfusion, easily resulting in CNS complications. In the study conducted by scholars Kanthasamy et al, it was shown that unbalanced induction of general anesthesia would further aggravate patients' stress reaction, lead to more significant hemodynamic fluctuations, and cause obvious impact on patients' cerebral circulation [22]. The American Stroke Association noted that blood pressure is an important factor affecting the occurrence of stroke and that changes in perioperative blood pressure also affect the cerebral circulation to some extent, increasing the possibility of postoperative cerebrovascular accidents [23]. This study found that the incidence rate of cerebrovascular accidents was significantly higher in the general anesthesia group than in the nongeneral anesthesia group (*P* < 0.001), and at *T*_2_, *T*_3_, and *T*_4_, the HP and MAP were significantly different between the two groups (*P* < 0.05), proving that the hemodynamic fluctuations caused by general anesthesia were the main reason affecting cerebrovascular accidents.

Prior studies have shown that if the occurrence of cerebrovascular accidents was regarded as the only dependent variate and factors such as general anesthesia and number of anesthetic drugs were regarded as the independent variate, then BMI ≥23 kg/m^2^, number of anesthetic drugs ≥4, and intraoperative blood pressure ≥140 mmHg were also the risk factors affecting cerebrovascular accidents in hip fracture patients [24]. The association of BMI with cerebrovascular accidents lies in the fact that the diet of obese patients has an excessive amount of oil-containing components and that their obesity is aggravated by postoperative bed rest, but when general anesthesia is considered as a variate, body mass can also affect the amount of anesthetic drugs. The drugs used in general anesthesia for hip fracture patients are mainly cerebral vasoconstrictors, which are able to increase cerebrovascular resistance and affect cerebral blood flow, and greater dosage may cause higher risk of unexpected events. In addition, most studies did not demonstrate that age was related to cerebrovascular accidents [25], but according to the multiple logistic regression in this study, it was found that *P* < 0.05 at age ≥80 years, which might be explained by the fact that when general anesthesia was a factor to consider, the surgical risk coefficient was significantly higher in elderly patients; especially, those with preoperative multivisceral disease were more likely to trigger cardiovascular and cerebrovascular diseases, so under general anesthesia, age ≥80 years was also a risk factor causing the presence of general anesthesia. If the recovery time after general anesthesia of such patients exceeds 90 min, the involvement of anesthetic drugs, patients' preoperative comorbidities, vital organ failure, and other conditions should also be taken into consideration, and if the delay recovery cannot be explained after excluding all factors, it is necessary to speculate on the possibility of cerebrovascular accidents based on intraoperative blood pressure, heart rate fluctuation, and pupil changes and fully focus on the vital sign observation in the high-risk period to prevent cerebrovascular accidents.

To sum up, general anesthesia is a risk factor affecting the occurrence of cerebrovascular accidents in hip fracture patients, and age ≥80 years, BMI ≥23 kg/m^2^, number of anesthetic drugs ≥4, intraoperative blood pressure ≥140 mmHg, and intraoperative heart rate ≥80 bpm will further increase the possibility of cerebrovascular accidents.

## Figures and Tables

**Figure 1:** Comparison of incidence rates of cerebrovascular accidents in patients (*n* (%)). Note: the black areas indicated cerebrovascular accidents, and the gray areas indicated no cerebrovascular accidents; (a) the general anesthesia group and (b) the nongeneral anesthesia group. In the general anesthesia group, there were 34 patients who had cerebrovascular accidents (28.3%) and 86 patients who had no cerebrovascular accidents (71.6%); and in the nongeneral anesthesia group, there were 6 patients who had cerebrovascular accidents (5.0%), and 114 patients had no cerebrovascular accidents (95.0%).

**Figure 2:** Comparison of changes in patients' hemodynamic indicators ($\bar{x}$ ± *s*). Note: the horizontal axes from left to right indicated *T*_1_, *T*_2_, *T*_3_, and *T*_4_, the lines with dots indicated the general anesthesia group, and the lines with blocks indicated the nongeneral anesthesia group; # indicated *P* < 0.05.

**Table 1:** Comparison of patients' general information.

Group	General anesthesia group (*n* = 120)	Nongeneral anesthesia group (*n* = 120)	*X* ^2^/*t*	*P*
Gender			0.068	0.794
Male	50	52		
Female	70	68		
Age (years)				
Range	64–86	64–88		
Mean age	76.98 ± 2.68	76.96 ± 2.58	0.059	0.953
Mean body mass (kg)	64.21 ± 2.14	64.23 ± 2.65	0.064	0.949
BMI (kg/m^2^)	22.68 ± 2.54	22.72 ± 2.45	0.124	0.901
Marital status			0.081	0.776
Married	84	86		
Unmarried/divorced/widowed	36	34		
Complications				
Hypertension	35	36	0.020	0.888
Diabetes	38	36	0.078	0.780
Cerebrovascular accidents			0.084	0.772
Yes	34	32		
No	86	88		
Place of residence			0.067	0.796
Urban area	66	64		
Rural area	54	56		
Monthly income (yuan)			0.068	0.795
≥4000	68	66		
<4000	52	54		
Living habit				
Smoking history	42	44	0.073	0.788
Drinking history	52	50	0.068	0.794
Educational degree			0.308	0.579
Senior high school and below	84	80		
College and above	36	40		

**Table 2:** Association between general anesthesia and the occurrence of cerebrovascular accidents.

Factor	*B*	SE	Wald	*P*	OR (95% CI)
General anesthesia	1.598	0.496	9.924	0.001	1.812 (1.812–12.684)

**Table 3:** Multivariate analysis on cerebrovascular accidents in hip fracture patients under general anesthesia.

Factor	*B*	SE	Wald	*P*	OR (95% CI)
Age ≥80 years	1.486	0.488	9.561	0.003	4.362 (1.712–11.120)
BMI ≥23 kg/m^2^	1.068	0.510	4.687	0.035	2.980 (1.123–7.985)
Number of anesthetic drugs ≥4	1.221	0.458	7.468	0.001	3.368 (1.423–8.136)
Intraoperative blood pressure ≥140 mmHg	1.678	0.465	12.986	<0.001	5.214 (2.214–12.985)
Intraoperative heart rate ≥80 bpm	1.468	0.464	9.935	0.002	4.356 (1.798–10.985)

## Data Availability

The data used to support the findings of this study are available from the corresponding author upon reasonable request.
